This article has been retracted.

# Effect of New Nursing on Patients with Acute Cerebral Infarction

**DOI:** 10.1155/2022/1863129

**Published:** 2022-05-02

**Authors:** Shengqin Gu, Xiaomei Gao, Wei Gu, Mulei Jiang, Dongmei Qi

**Affiliations:** ^1^Department of Encephalopathy, Nanjing Pukou Hospital of Traditional Chinese Medicine, 211800 Nanjing City, Jiangsu Province, China; ^2^Department of Nursing, Nanjing Pukou Hospital of Traditional Chinese Medicine, 211800 Nanjing City, Jiangsu Province, China

## Abstract

**Objective:**

To explore the effect of the comfortable intervention-based nursing mode under the quality nursing intervention combined with Internet mobile health on the quality of life (QOL) and psychological status of patients with acute cerebral infarction (ACI).

**Methods:**

90 ACI patients treated in our hospital (June 2019-June 2020) were chosen and equally split into the experimental group (EG) and control group (CG) according to the order of admission. CG received routine nursing, while EG received the comfortable intervention-based nursing mode under the quality nursing intervention combined with Internet mobile health to compare the clinical indexes between the two groups.

**Results:**

Compared with CG, EG after intervention achieved obviously higher SS-QOL, ESCA, and GCQ scores (*P* < 0.001), and lower MSSNS and NIHSS scores (*P* < 0.001).

**Conclusion:**

The application of the comfortable intervention-based nursing mode under the quality nursing intervention combined with Internet mobile health effectively improves QOL and alleviates the negative emotions of patients. Compared with routine nursing, this model has higher application value, and further research of the joint intervention will help build better a solution for patients.

## 1. Introduction

Cerebral infarction (CI), also known as ischemic stroke, refers to the insufficient blood supply to the brain or circulation disorders caused by various reasons, resulting in cerebral hypoxia and ischemia [1, 2]. The clinical symptoms of the disease vary, in which mild patients may have no symptoms, recurrent vertigo, or limb paralysis, while the severe ones may not only have limb paralysis but also have acute coma and death [3]. Smoking and drinking are high-risk predisposing factors of CI, and basic diseases such as hyperlipidemia, heart disease, and hypertension are also the causes of CI. At the same time, the disease often occurs in the elderly and patients with hypertension and coronary heart disease. Relevant literature indicates that CI, the second leading cause of global death and the primary cause of disability or death in Chinese residents, has increasing prevalence, incidence, and mortality both in developing and developed countries, seriously affecting people's life safety [4]. According to relevant literature, the number of deaths from stroke worldwide in 2017 was 5.9 million per year, while epidemiological surveys have revealed that stroke has become the main cause of death in China, constituting the three main causes of human death together with malignant tumors and heart diseases [5, 6]. Çelebi et al. [7] have pointed out that about 2.39 million people suffer from stroke every year, of which ischemic stroke accounts for 75%. Shams et al. [8] have noted that about 69% of patients with acute cerebral infarction (ACI) experience a significant increase in blood pressure within 24 h after admission due to inadequate control of hypertension before stroke or increased intracranial pressure, poststroke stress response, and autonomic nerve dysfunction. This early increase in blood pressure, also known as acute hypertension response, has a short reaction time, and most patients can return to the normal blood pressure level before stroke within 7 days after onset. The response is closely related to poor prognosis and nursing measures, so implementing efficient nursing measures for ACI patients is of great significance to improve the prognosis [9].

Although routine nursing has a certain nursing effect, it is a nursing model developed based on traditional experience that lacks scientific evidence, and its appropriateness, scientificity, and effectiveness are hard to be judged [10]. With the progress of medical technology and the rapid development of the Internet, Internet mobile health has gradually become the focus of attention. The application of Internet mobile health, especially telemedicine for ACI patients, can be regarded as the enhancement of self-care. It can enable ACI patients to complete diet and blood pressure data in real time through the Internet, thus further realizing the establishment of electronic health records, interactive education, remote monitoring, and online discussion, which is conducive to building a sustainable and stable doctor-patient relationship [11]. Meanwhile, based on the people-oriented concept, the comfortable intervention-based nursing mode under the quality nursing intervention can effectively meet the nursing needs of patients and further enhance their quality of life (QOL). In addition, it has been confirmed that Internet mobile health has a remarkable effect on the management of chronic diseases such as hypertension [12]. However, more studies have also revealed that this nursing mode can promote the QOL of stroke patients [13]. However, the intervention of this nursing model combined with Internet mobile health is rarely reported. Therefore, this paper carried out the joint intervention on the subjects to provide more clinical evidence-based proof for ACI patients.

## 2. Material and Methods

### 2.1. General Information

The 90 ACI patients treated in our hospital (June 2019-June 2020) were chosen as the study subjects and equally split into experimental group (EG) and control group (CG) according to the order of admission. This study conformed to the Declaration of Helsinki (2013) [14].

### 2.2. Recruitment of Subjects

#### 2.2.1. Inclusion Criteria

(1) Patients met the diagnostic criteria of ACI in the Sixth National Academic Conference on Cerebrovascular Diseases [15] and were confirmed by brain MRI and CT, with the clinical manifestations including aphasia, disturbance of consciousness, and brain edema; (2) the admission time after onset was less than 72 h; (3) patients had no communication barriers; (4) patients had no serious dysfunctions in the heart, liver, and kidney, or other serious diseases such as malignant tumors; (4) patients had the first onset; and (6) the patients were aged more than 45 years.

#### 2.2.2. Exclusion Criteria

(1) Patients with a definite history of dementia or cognitive impairment; (2) patients in the active phase of chronic infectious diseases or those with acute infectious diseases; (3) patients with intracranial tumor lesions; (4) patients with hemiplegia or muscle strength of the affected limb > grade 3; (5) patients with audiovisual impairment and those who could not cooperate with the researchers; and (6) patients participating in other trials.

### 2.3. Methods

#### 2.3.1. CG

EG received routine nursing, including basic nursing, medication guidance, health education, and dietary intervention. Meanwhile, the vital indexes of patients were monitored, and effective treatment measures were taken if any abnormalities occurred.

#### 2.3.2. EG

*(1) Comfortable Intervention-Based Nursing Mode under the Quality Nursing Intervention*. (1) Environmental comfortable nursing. When carrying out nursing services, medical staff paid attention to the living environment of ACI patients, regularly disinfected the wards, and maintained the wards clean. At the same time, the temperature of the wards was appropriately controlled at 19°C-27°C. The windows were regularly opened for ventilation to ensure fresh air in the wards, and the humidity of the wards was adjusted to 55%-65%. The patients were allowed to put appropriate personal things in the wards, such as family photos and crafts, to increase the family atmosphere and reduce their psychological pressure. Medical staff also placed flowers and green plants to add vitality in the wards, so that patients could keep a cheerful and pleasant state of mind. (2) Physiological comfortable nursing. Medical and nursing staff needed to help patients with inconvenient behaviors to change their positions, and massaged the compressed parts of limbs to promote local blood circulation and avoid the occurrence of pressure sores. At the same time, the painless puncture technique was used to implement infusion nursing for patients. After the patients' condition was stable, patients were massaged to facilitate rapid recovery. Finally, based on the patients' self-care ability, illness, and awareness, medical staff needed to help patients maintain good hygiene and improve their comfort. For example, hydrogen peroxide was used for the oral wiping of patients to reduce the overgrowth of oral bacteria and decrease the incidence of infection and oral ulcers. (3) Psychological comfortable nursing. CI patients had various negative emotions, such as depression, anxiety, and pessimism. When carrying out nursing work, medical staff should adopt a cordial and mild attitude to communicate with patients and timely feedback their emotional expression, regularly carry out health education, explain CI-related knowledge and precautions to them, and encourage them to actively adjust the negative emotions. The patients were instructed to watch videos and listen to music to divert their attention when depression occurred. If they had serious signs of psychological crisis, nursing staff should timely provide them with psychological counseling while maintaining a kind and friendly attitude to reduce their resistance and gain their trust. (4) Dietary comfortable nursing. Due to an older age, ACI patients often had a higher blood pressure level compared with normal people, and most patients were complicated with diseases such as declined gastrointestinal function. Therefore, medical staff should formulate reasonable diet plans, mainly including high vitamin and protein without stimulating foods, based on the condition, personal preferences, and nutritional requirements of the patients.

*(2) Internet Mobile Health*. Guided by the nursing staff, the patients downloaded *Cardio-Cerebrovascular Steward* APP and entered the patient interface after real-name authentication. At the same time, nursing staff instructed the patients to skillfully use APP and established electronic files of the disease and basic information. In addition, the nursing staff trained the patients to measure the body indicators skillfully and upload the data regularly. The patients uploaded data such as blood pressure and heart rate once a day and tried to upload data such as medication, diet, and body weight every three days to the *Cardio-Cerebrovascular Steward* APP. Those who failed to timely upload data would be reminded by the WeChat client in time. Medical staff needed to carry out timely analysis after collecting the data of patients, remotely monitor patient blood pressure, develop personalized nursing and treatment plans based on their physical condition, and adjust the management plans and medication according to their disease condition. Patients were given health education through APP and WeChat, supplemented by publicity materials on CI knowledge. The nursing staff regularly used the management terminal of the *Cardio-Cerebrovascular Steward* APP to push the knowledge related to disease or health to patients, including general knowledge of healthy life, disease management, and rational medication in the forms of knowledge classroom, short videos, and pictures to enhance the accumulation of health knowledge of patients and improve their interest in autonomous learning.

### 2.4. Observation Indexes

The *Stroke-Specific Quality of Life Stroke (SS-QOL)* scale [16] was adopted to evaluate the QOL of both groups after intervention, with a total of 49 items covering 12 domains of energy, family role, language, activity, emotion, personality, psychological ability, social role, thinking, upper limb function, vision, and work/labor. Each item scored 0-5 points and a higher score suggested higher QOL.

The *Mental Status Scale in Nonpsychiatric Settings (MSSNS)* scale [17] was used to evaluate the overall psychological status of patients after intervention, including a total of 38 items scored by the four-point method, with 1 point as “no or few,” 2 points as “sometimes,” 3 points as “often,” and 4 points as “mostly.” A higher score indicated higher intensity of emotional response.

The *Exercise of Self-Care Agency Scale (ESCA)* [18] was applied to evaluate the self-care ability of patients after intervention, including four aspects of self-concept (items 1-8), self-responsibility (items 9-14), self-care skills (items 15-26), and health knowledge (items 27-43), with each aspect scoring 4 points. A higher score denoted higher self-care ability of patients.

The neurological function of both groups after the intervention was measured using the *National Institute of Health Stroke Scale (NIHSS)* [19], with 11 items and a total score of 42 points. A higher score represented more severe neurological impairment in patients.

The degree of comfort in both groups was assessed using Kolcaba's *General Comfort Questionnaire (GCQ)* [20], including physical, psychological, spiritual, sociocultural, and environmental dimensions, with a total of 28 items. The items were scored by a 1-4 Likert scoring method, with 1 point as “strongly disagree” and 4 as “totally agree.” For inverse questions, 1 point indicated “totally agree” and 4 points denoted “strongly disagree.” A higher score represented more comfort.

### 2.5. Statistical Treatment

In this study, the data were processed by software SPSS 20.0 and graphed by GraphPad Prism 7 (GraphPad Software, San Diego, USA). The study included enumeration data and measurement data, tested by *x*^2^, *t* test, and normality test. When *P* < 0.05, the differences were statistically significant.

## 3. Result and Analysis

### 3.1. Comparison of Baseline Data

No remarkable difference was observed in gender, age, BMI, onset time, complications, occupation, education, religion, family income, and residence between the two groups (*P* > 0.05), as presented in Table 1.

### 3.2. Comparison of SS-QOL Scores after Intervention

The SS-QOL score was remarkably higher in EG than in CG after intervention (*P* < 0.001). See Figure 1.

### 3.3. Comparison of MSSNS Scores after Intervention

Table 2 shows a lower MSSNS score in EG than in CG (*P* < 0.001).

### 3.4. Comparison of ESCA Scores after Intervention

The ESCA score in EG was obviously higher than that in CG after intervention (*P* < 0.05), as detailed in Table 3.

### 3.5. Comparison of NIHSS Scores after Intervention

Figure 2 demonstrates a lower NIHSS score in EG than in CG after intervention (*P* < 0.001).

### 3.6. Comparison of GCQ Scores after Intervention

The GCQ score in EG was markedly higher than that in CG after intervention (*P* < 0.001). See Table 4.

## 4. Discussion

ACI is common in clinical practice, and patients often show symptoms such as vertigo and headache and even language and motor dysfunctions in severe cases. Meanwhile, continuous aggravation of the disease will endanger the life safety of patients. Raychev et al. [21] have pointed out that only 9% of CI patients can be completely cured after symptomatic treatment, and most patients experience sequelae after treatment, which not only affects the recovery of the disease but also further increases the physical and mental pressure of the patients. Relevant literature has confirmed that efficient nursing intervention for ACI patients can effectively boost the rehabilitation effect [22]. Routine nursing mode can only provide the patients with nursing services within the regulations, failing to meet their request for diversified nursing. When patients receive nursing passively, they can easily have negative emotions because their needs are unmet, leading to more doctor-patient disputes. The comfortable intervention-based nursing mode under the quality nursing intervention is a newly applied nursing mode that has gained clinical recognition. Following the people-oriented principle, this patient-centered nursing model provides comprehensive and meticulous nursing services for patients. Compared with routine nursing, the comfortable intervention-based nursing mode under the quality nursing intervention is more standardized, systematic, and comprehensive. According to related literature, most patients are unfamiliar with the hospital environment and have limited knowledge about the disease, which leads to negative emotions such as fear, anxiety and depression. Some patients even lose treatment confidence with reduced compliance, affecting the overall therapeutic effect [23]. In the comfortable intervention-based nursing mode under the quality nursing intervention, medical staff formulate reasonable nursing programs according to the psychological demands of patients and create a comfortable and harmonious treatment environment for them, ultimately achieving the purpose of satisfying patients and treating diseases. In addition, the rapid development of the Internet has also led to the diversified development of medical care. The application of the Internet mobile client enables medical staff to understand the condition of patients in real time and also comprehensively record the health records of CI patients, so that doctors can search, classify, and collect the patient information. Naoki et al. [24] carried out a series of randomized controlled trials and found that Internet mobile health effectively improved the blood glucose level and self-management ability of patients with type 2 diabetes and enhanced their QOL, confirming the remarkable application effect of Internet mobile health in clinical nursing. In this study, the SS-QOL score was higher in EC after intervention compared with CG (*P* < 0.001), indicating that the comfortable intervention-based nursing mode under the quality nursing intervention combined with Internet mobile health has a significant effect on improving the QOL of ACI patients. In addition, the comfortable intervention-based nursing mode under the quality nursing intervention focuses on patients' feelings during hospitalization and requires nursing staff to notice the nursing details, so that patients feel humanistic care with better self-care ability. The application of this nursing model for ACI patients can scientifically evaluate their psychological state and popularize the relevant knowledge to them, which enables them to correctly understand the disease, rationally and calmly cooperate with the treatment of hospitals, establish confidence in combating the disease, and strive for early recovery. Based on this nursing model, the introduction of Internet mobile health can effectively improve the psychological state of patients and enhance their self-care ability. This is because Internet mobile health enables medical staff to communicate with patients anytime, through which patients can timely feedback the disease condition and doctors can provide emergency and rescue services in time. Moreover, since patients regularly upload the data of the body indexes daily, medical staff can adjust the nursing plans in real time and provide individual nursing measures, thereby effectively saving hospital resources and reducing medical costs.

NIHSS is mainly adopted to assess the improvement of neurological impairment in patients, while it also reflects the recovery of neurological function. Both groups received nursing services, but the NIHSS score in EG was lower after intervention (*P* < 0.001), fully confirming the clinical advantages of the comfortable intervention-based nursing mode under the quality nursing intervention combined with Internet mobile health, which is consistent with the report of Mutsumi et al. [25]. In addition, this study also showed that the GCQ score after intervention was remarkably higher in EG than in CG (*P* < 0.001), indicating that compared with routine nursing, the comfortable intervention-based nursing mode under the quality nursing intervention can effectively improve the comfort and the prognosis of patients. This study has some inadequacies. (1) Clinical evaluation was carried out through scales. When patients answered questions, a certain degree of subjectivity and willfulness was inevitable, which affected the final results of the clinical trials to some extent. (2) The intervention time was short and the source of cases was single because the selected cases in this study were all patients treated in local hospitals. (3) Due to the limitation of the observation period, the clinical study failed to include enough samples, resulting in biased results. Therefore, in the future, the study design should be improved with loner follow-up time to thoroughly and meticulously explore the nursing effect of the comfortable intervention-based nursing mode under the quality nursing intervention combined with Internet mobile health on ACI patients from multiple perspectives. To sum up, the preliminary conclusion of this study still needs to be refined by more subsequent studies.

## 5. Conclusion

In conclusion, the comfortable intervention-based nursing mode under the quality nursing intervention combined with Internet mobile health can effectively enhance QOL, improve the brain nerve function, and alleviate the psychological state of ACI patients. In recent years, the wide application of Internet mobile health has also led to the diversified development of clinical nursing modes, which opens up a new direction for clinical nursing pathways and promotes the comprehensive and systematic development of nursing for ACI patients.

## Figures and Tables

**Figure 1:** Comparison of SS-QOL scores after intervention ($\overset{¯}{x}\pm s$). Note: the abscissa represented EG and CG, and the ordinate represented the SS-QOL score (points). The SS-QOL scores of EG and CG were 208.96 ± 12.73 and 160.16 ± 11.41. ∗ indicated a notable difference in the SS-QOL scores between the two groups after intervention (*t* = 19.149, *P* < 0.001).

**Figure 2:** Comparison of NIHSS scores after intervention ($\overset{¯}{x}\pm s$). Note: The abscissa represented EG and CG, and the ordinate represented the NIHSS score (points). The NIHSS scores of EG and CG were 8.93 ± 1.94 and 20.33 ± 2.75. ∗ indicated a notable difference in the NIHSS scores between the two groups after intervention (*t* = 22.723, *P* < 0.001).

**Table 1:** Comparison of baseline data.

Items	EG (*n* = 45)	CG (*n* = 45)	*x* ^2^/*t*	*P*
Gender			0.046	0.830
Male	27 (62.22%)	26 (60.00%)		
Female	18 (37.78%)	19 (40.00%)		
Age ($\;\overset{¯}{x}\pm s$, yrs)	59.11 ± 8.85	61.82 ± 9.46	1.403	0.164
BMI (kg/m^2^)	20.63 ± 0.74	20.75 ± 0.66	0.812	0.419
Onset time (h)	12.93 ± 7.59	13.87 ± 7.13	0.606	0.546
Complications				
Hypertension	17 (37.78%)	18 (40.00%)	0.047	0.829
Diabetes	16 (35.56%)	16 (35.56%)	0.000	1.000
Hyperlipidemia	12 (26.67%)	11 (24.44%)	0.058	0.809
Occupation				
Civil servants				
Teachers	15 (33.33%)	14 (31.11%)	0.059	0.822
Financial staff	14 (31.11%)	16 (35.56%)	0.200	0.655
Other	16 (35.56%)	15 (33.33%)	0.049	0.824
Education				
Primary and junior high school	15 (33.33%)	16 (35.56%)	0.049	0.824
High school and junior college	17 (37.78%)	16 (35.56%)	0.048	0.827
University and above	13 (28.89%)	13 (28.89%)	0.000	1.000
Religion			0.067	0.796
Yes	10 (22.22%)	9 (20.00%)		
No	31 (77.78%)	36 (80.00%)		
Family income			0.067	0.796
≥3000 yuan/(month·person)	35 (77.78%)	36 (80.00%)		
<3000 yuan/(month·person)	10 (22.22%)	9 (20.00%)		
Residence			0.048	0.827
Urban area	28 (62.22%)	29 (64.44%)		
Rural area	17 (37.78%)	16 (35.56%)		

**Table 2:** Comparison of MSSNS scores after intervention ($\overset{¯}{x}\pm s$).

Group	*n*	MSSNS score
EG	45	44.41 ± 2.63
CG	45	66.08 ± 2.75
*t*		38.202
*P*		<0.001

**Table 3:** Comparison of ESCA scores after intervention ($\overset{¯}{x}\pm s$).

Group	*n*	Self-concept	Self-responsibility	Self-care skills	Health knowledge
EG	45	3.08 ± 0.28	2.36 ± 0.31	2.68 ± 0.21	3.07 ± 0.19
CG	45	1.52 ± 0.19	1.14 ± 0.14	1.08 ± 0.13	1.34 ± 0.27
*t*		30.926	24.060	43.457	35.151
*P*		<0.001	<0.001	<0.001	<0.001

**Table 4:** Comparison of MSSNS scores after intervention ($\overset{¯}{x}\pm s$).

Group	*n*	GCQ score
EG	45	65.16 ± 3.21
CG	45	45.38 ± 2.76
*t*		31.343
*P*		<0.001

## Data Availability

Data to support the findings of this study is available on reasonable request from the corresponding author.
